The article "Study on Discrete Dynamic Modeling of College Students' Innovative Employment Security Mechanism under the Environment of Internet of Things" was published in 2022. Journal: Comput Intell Neurosci.

# Study on Discrete Dynamic Modeling of College Students' Innovative Employment Security Mechanism under the Environment of Internet of Things

**DOI:** 10.1155/2022/4637180

**Published:** 2022-04-15

**Authors:** Liming Gu, Xue Chen

**Affiliations:** ^1^Chengdu Normal University, Chengdu, 610000, Sichuan, China; ^2^Chengdu Experimental School, Chengdu, 610000, Sichuan, China

## Abstract

The innovative mechanism of college students' employment security is a series of security measures implemented by the state and society to solve the mismatch between the scale growth of college graduates and the jobs provided by the society. In order to promote the development of emerging Internet of things technologies, users can find interesting and valuable information from a large number of data sets and use this information to meet the needs of users. This article mainly studies the historical development trend and discrete dynamic modeling and analysis technology of college students' innovative employment security mechanism under the environment of Internet of things. Using two different modeling methods of Bayesian network and BP neural network, this article makes discrete dynamic modeling on the influencing factors and employment security mechanism of college students' employment, so as to improve the college biological network innovation employment security mechanism and better help college students' employment.

## 1. Introduction

China has the largest number of college graduates in the world. The scale of higher education in China is unmatched by any other country, and the number of colleges and universities is in the forefront of all countries. However, the increase in the number of college students not only brings great opportunities and talent dividends to the country but also brings a series of challenges and social problems, the most important of which is the employment of graduates. The number of college students is growing, but the employment cannot match the growth rate of college students, resulting in a considerable number of graduates facing the dilemma of unemployment once graduation, and the “lying flat” and “gnawing the old” are growing day by day. At the same time, although some college students find jobs, they cannot give full play to their professional strengths, and the post functions do not match the skills they master Tengrong [1]. In view of the above situation, the Chinese government has paid full attention to it, adopted a series of employment security measures for college students, and adopted different and flexible assistance policies for different implementation objects, such as students, universities, and enterprises Kurszewska et al. [2].

In recent years, with the continuous development of computer, Internet, Internet of things, and various new sensors, information and data circulating in various fields have attracted more and more attention from all walks of life Zhang [3]. Nowadays, the way of data generation extends to all fields of society. Almost everything will produce information data, and these information data are finally collected and counted to form a huge data set, referred to as “big data” Pang et al. [4]. It mainly refers to the data set whose data scale exceeds that obtained, saved, and processed by traditional data management software. It can analyze and process big data, collect and extract from massive and scattered data, so as to obtain valuable information for users, and then conduct discrete dynamic modeling to associate with college students' employment security Zhu [5]. Discrete dynamic modeling technology is also very practical. It is suitable for most fields and belongs to a comprehensive cutting-edge technology. With the continuous exploration and promotion of personnel in various fields, the technology has made great progress and has been successfully applied in various fields Pirbhulal et al. [6]. For example, the e-commerce platform uses the user search and browsing record data to recommend the products that users expect to buy, establish relevant models, and promote user consumption. The public security system uses all the monitoring data to obtain all kinds of information of the suspect, master its whereabouts, and make the big data play a major role in the reconnaissance work Cui [7].

This article mainly consists of three parts. The first part introduces the development status of University Biological Networking Innovation and employment security mechanism and discrete dynamic modeling algorithm. The second part analyzes the application of discrete dynamic modeling method in employment security mechanism under the background of Internet of things and puts forward scientific and reasonable suggestions by combining Bayesian network algorithm, grey analysis method, and BP neural network with today's College Students' employment security system. The third part analyzes and compares the research results, establishes relevant discrete dynamic models, finds out the hidden relationship between the calculation data and the employment security mechanism and the employment status of college students, and puts forward effective suggestions to improve the security mechanism.

## 2. Related Work

The concept of big data has long been mentioned. As early as the last century, Toffler, a futurist, mentioned the word “big data” in his works Tang et al. [8]. At the beginning of this century, analysts pointed out that the number of big data of the group is diverse. McKinsey formally defined the concept of big data Wang et al. [9]. After that, the United States released a report on big data Internet of things analysis technology, marking that big data Internet of things analysis and processing technology has become a technology at the level of national science and technology strategy Zhang et al. [10]. Since then, the development and maturity of computer, Internet, and other technologies have provided fertile ground for the seeds of big data Internet of things analysis technology to thrive.

The United States is the first country to upgrade the discrete dynamic modeling technology from the civil field to the national strategic level. Through the “three-step” plan, it has formed a technology leader ahead of other countries in various fields in the country Liu et al. [11]. The “three-step” plan mainly includes the following contents: first, accelerate the research of discrete dynamic modeling and analysis technology and realize the application of discrete dynamic modeling and analysis in some fields of the Internet of things Zhang and Liu [12]. Then, aiming at the derivative problems brought by discrete dynamic modeling technology, a series of regulations are implemented. Finally, strengthen the construction of discrete dynamic modeling production system to enhance the country's competitiveness in the field of data analysis.

On the development of discrete dynamic modeling and analysis technology, Britain has absorbed the valuable experience of the United States. According to the needs of the country and the people, strengthen the investment in data research and development and focus on the application of Internet of things analysis in advanced fields Pu [13]. In addition, the UK government strongly advocates digital strategy to improve the employment problem in the country.

As a neighbor of China, South Korea has the world's leading network transmission speed and the popularity of intelligent devices, which also brings its inherent advantages in the development of the Internet of things Meng et al. [14]. Under the policy of “creative economy,” various departments of the Korean government cooperate to speed up the development of discrete dynamic modeling and analysis technology. By 2016, South Korea had introduced a policy based on discrete dynamic modeling technology to meet the opportunities and challenges brought by global digitization.

China also focuses on developing discrete dynamic modeling technology. At the Fifth Plenary Session of the 18th CPC Central Committee, the government took the development of big data Internet of things as a national strategy Shumin and Liu [15]. The Ministry of industry and information technology has also formulated an industrial development plan for the development of discrete dynamic modeling and made different policy arrangements for different periods.

The above is the development history of discrete dynamic modeling analysis and processing technology and its development status in various countries.

## 3. Methodology

### 3.1. Model Construction of Bayesian Network Algorithm in College Students' Innovative Employment Security Mechanism

The original method can only understand the impact of policies through simple manual prediction and actual implementation. Nowadays, the vigorous development of Internet of things analysis technology provides us with new research methods. In the process of proposing and applying the innovative employment security mechanism for college students, it is necessary to consider the role, influence, and effectiveness of the corresponding security mechanism after practical application.

We can use the Internet of things technology. The security mechanism is to collect and analyze the employment information of college students after the implementation of the employment security mechanism and the employment information that does not enjoy the security and carry out dynamic data prediction modeling, so as to infer the weight of the impact of different college students' employment security mechanisms on the employment situation and improve the effectiveness of the employment security mechanism. This article uses Bayesian network algorithm to predict and analyze the security mechanism of College Students' innovative employment. Before that, the Bayesian theorem is briefly introduced, mainly including the following concepts:

(1) Random test
Random test refers to the test that cannot know all the results in advance before the event occurs. All the results obtained from the random test constitute the sample space Ω of the test. The sample space contains all events.
(2) Probability
The probability of occurrence of event X in the sample space is called probability, and the value is *p* (*x*). The probability satisfies the following conditions:
  (1) $$\begin{array}{c} P\left(\Omega \right)=1,\\ P\left(X\right)\geq 0,\\ P\left(X\cup Y\right)=P\left(X\right)+P\left(Y\right),\;X\cap Y=\emptyset . \end{array}$$
(3) Joint probability
The combination probability that contains all multiple random variables and satisfies their respective probabilities. For multiple random variables, the joint probability is
  (2) $$\begin{array}{c} P\left(X_{1},\ldots ,X_{n}\right), \end{array}$$
of which
  (3) $$\begin{array}{c} \sum_{X_{1},\ldots ,X_{n}}X_{1},\ldots ,X_{n}=1. \end{array}$$
(4) Conditional probability refers to the probability that event *x* occurs under the condition that event *y* has occurred, which can be expressed as
  (4) $$\begin{array}{c} P\left(X|Y\right)=\frac{P\left(X,Y\right)}{P\left(Y\right)}. \end{array}$$
(5) Bayesian theorem:

(5) $$\begin{array}{c} P\left(Yi|X\right)=\frac{P\left(X,Yi\right)}{P\left(X\right)}\\ =\frac{P\left(Yi\right)P\left(X|Yi\right)}{\sum_{i=1}^{n}P\left(Yi\right)P\left(X|Yi\right)}. \end{array}$$

Bayesian theorem can obtain unknown posterior probability through the determined prior probability. When you cannot determine the probability of an event, you can use the probability of other related events to infer the probability of the event.

Bayesian network is mainly composed of (*X*, *A*, ∅). The first two parts (*X*, *A*) is a directed acyclic graph structure, and *X* is the set of nodes in Bayesian network. These sets can be observable variables, hidden variables, or unknown variables. Two variables with causality will produce a directed arrow connecting two nodes. After the two nodes are connected with each other, the conditional probability values of the two nodes can be obtained. *A* is the set of arrows in the network.

The following figure is a common Bayesian network diagram.

The structure diagram of Bayesian network is shown in Figure 1. In the figure, the one issuing the arrow is called the parent node, and the arrow refers to the child node. For example, a is the parent node of B. A parent node can have multiple child nodes, and a child node can also have multiple parent nodes. The arrow represents that the two are interrelated. Therefore, through Bayesian network, we can deduce a and *h* from C, or C from a and H.

*X* is the set of nodes in Bayesian network, which can be observable variables, hidden variables, or unknown variables. Two variables with causality will produce a directed arrow connecting two nodes. After the two nodes are connected with each other, the conditional probability values of the two nodes can be obtained. *A* is the collection of arrows in the network.

Conditional independence has been assumed in Bayesian networks, that is, a parent node is given, which will be independent of all its nondescendant nodes. Therefore, the joint probability of all nodes in Bayesian network is the product of the conditional probability of each node.

(6) $$\begin{array}{c} P\left(X_{1},\ldots ,X_{n}\right)=\overset{n}{\underset{i=1}{\prod }}P\left(Xi|X_{1},\ldots ,X_{n}\right)\\ =\overset{n}{\underset{i=1}{\prod }}P\left(Xi|\pi \left(Xi\right)\right). \end{array}$$

Therefore, as long as the directed graph model of Bayesian network is constructed, the relationship between each node can be obtained, and then, the probability distribution of nodes can be obtained by determining the parameter ø.

According to the Bayesian network algorithm, we can build a structure diagram, mark the end node as employed and unemployed college students, and its related parent node can be set as individual information of college students, such as gender, education, and skills. Then, according to the collected employment information of college students in a certain year in a certain region and the probability of different security mechanisms to help college students obtain employment, the data are input into the model. Through this model, we can obtain the relationship between graduates' employment and employment security policy and individual factors, so as to get the rated relationship between them.

### 3.2. BP Neural Network Combined with Discrete Dynamic Modeling of Internet of Things to Construct the Evaluation Model of College Students' Innovative Employment Security Mechanism

With the continuous expansion of the scale of college graduates, it is particularly important to innovate the employment security mechanism to alleviate the employment pressure of college students. How to find the mechanism with the highest quality and the best effect among many security mechanisms is related to the optimization and structural adjustment of employment security mechanism.

There are many quality evaluation models of employment security mechanism, which can be roughly divided into the following three categories: subjective evaluation model, objective evaluation model, and subjective and objective evaluation model. Among them, the subjective evaluation model is the evaluation of College Students' innovative employment security mechanism by professional researchers in this field. This approach often varies widely in terms of results, personal feelings, and persuasion. The objective evaluation model uses this algorithm to evaluate the innovative employment security mechanism of college students. This method does not include personal subjective views, and all evaluation results depend on input parameters. Compared with the subjective evaluation model, the evaluation effect of this model is better. However, the goal model often uses only one algorithm, and the employment security mechanism of college students is composed of a variety of security measures. A single algorithm is difficult to reflect the quality evaluation of all mechanisms. The third subjective and objective evaluation model combines the advantages of the first two evaluation models and has high evaluation accuracy, but at the same time, the modeling speed of the model is the slowest and the efficiency is the lowest.

In order to evaluate the quality of college students' innovative employment security mechanism with higher accuracy and efficiency, this article uses BP neural network method to build a model and analyze its evaluation effect.

BP neural network is a popular and mature algorithm. The principle is to carry out forward propagation after inputting data. If the expected result cannot be obtained in the output layer, the error will be propagated back to the input layer and the weight of neurons will be adjusted to repeat continuously to obtain the expected result.

This article combines the two analysis methods to evaluate the employment security mechanism of college students. The main steps are as follows:

Firstly, collect the employment data of college students and the data of employment security mechanism, preprocess the data, eliminate some wrong information, construct the corresponding model using grey analysis method and BP neural network algorithm, obtain the employment rate data of college students under different employment security mechanisms, and then adjust their weights by linear regression, Finally, the optimal evaluation model of college students' employment security mechanism is obtained, and the flow chart is shown in the figure below.

As shown in Figure 2, there are two methods to build the model of college students' employment security mechanism. First, preprocess the collected data and eliminate accidental data to reduce the error after analysis. There are four extracted feature vectors: employment area, salary, specialty matching, and working hours. These four features are respectively input into the neural network training mode for training to see whether the results meet the accuracy requirements. If the accuracy requirements are not met, the parameters are adjusted again and input into the neural network system for training. If the results meet the accuracy requirements, the characteristics that have the greatest impact on college students' employment will be output. After many experiments and simulations, it can be concluded that the salary has the greatest impact, and the other orders are region, working time, and major matching. Through this mechanism, we can put forward more reasonable suggestions on the employment security system of college students.

## 4. Result Analysis and Discussion

### 4.1. Bayesian Network Algorithm in College Students' Innovative Employment Security Mechanism Model Construction and Result Analysis

Finding new directions and ideas for college students' innovative employment through algorithm analysis is the development trend of big data of the Internet of things. The training sample set is constructed based on the data samples collected in recent years. Combined with the previous experience, the Bayesian network model can be constructed and the corresponding parameters can be obtained. If you have complete data, you can evaluate the Bayesian function by scoring and summing the obtained local data. At this time, the overall structure of Bayesian network will not be affected by this part of data. Therefore, we only calculate local data. For example, if random variables and training sets are defined respectively, the scoring function can be decomposed into

(7) $$\begin{array}{c} Sj=\sum_{i=0}^{m-1}wij\;xi+bj,\\ xj=f\left(Sj\right),\\ \text{score}\left(BN:D\right)=\overset{N}{\underset{i=1}{\sum }}\log\left(P_{BN}\left(X_{i}\right)-\frac{\log_{2}\;N}{2}\text{Dim}\left[G\right]\right). \end{array}$$

Through the above processing, we use two typical Bayesian networks. When the number of nodes is 8, the maximum number of node states is 2. When the training set is set to 1000, 2000, and 3000, the relationship between the data default rate can be obtained according to the time required for the algorithm to run, as shown in Figure 3.

It can be seen from the picture that when the default rate reaches 30%, the correlation between running time and the number of samples is almost negligible. In the graph of 1000 sample points, when the default rate is equal to 10, there is more than 1800 seconds of serial running time.

Through comparison, it is found that when using pl-em algorithm in Bayesian network, it can well reduce the communication overhead and is suitable for large sample learning. However, in the case of M nodes, the communication overhead will increase with the increase in the number of nodes, so the performance of this algorithm will be reduced.

Therefore, although pl-em algorithm is an effective method to learn Bayesian network, it also has great disadvantages. In particular, the huge amount of calculation required in the process of posterior probability calculation should be reasonably modified according to the selected inference engine.

When Bayesian network is used to deal with such uncertainty, it needs to be applied to the method of probability for reasoning. This method is also called Bayesian network calculation, that is, the posterior probability distribution *P* (*x*|*e*) is calculated using conditional probability. Bayesian network inference methods are divided into accurate inference and approximate inference, but it is proved that both methods are NP complete problems. Inference is carried out through the method of joint tree. The main principle is message passing using union tree.

The largest clique in the union tree determines the complexity of its reasoning, and it is also a core problem that we need to solve in Bayesian network using probability method. The triangulation operation of constructing the union tree can directly determine the size of the clique. Therefore, using the optimal triangulation operation can make the probability reasoning more accurate, and the order of BN's moral graph determines the optimal triangulation operation. Therefore, the root of making probability inference more accurate is to solve the optimal triangulation and find the optimal deletion ranking problem.

First build a union tree, then find the largest clique, and use VC to represent the variables in the clique to obtain the potential function of the clique:

(8) $$\begin{array}{c} \phi_{c}=\prod_{X\in Vc}P\left(X|pa\left(X\right)\right). \end{array}$$

Then, the potential function of the union tree is established as follows:

(9) $$\begin{array}{c} \phi_{JT}=\frac{\prod c\subset C\phi C}{\prod s\subset S\phi S}. \end{array}$$

The clique generated by the triangulation operation can represent the weight of the joint tree, and the weight of the above clique can be obtained as follows:

(10) $$\begin{array}{c} w\left(C\right)=\prod_{i=1}^{k}w\left(v_{i}\right). \end{array}$$

The operation tree weights are as follows:

(11) $$\begin{array}{c} w\left(JT\right)=\;\log_{2}\sum_{C}w\left(C\right). \end{array}$$

The main implementation of this algorithm is to convert BN into joint tree and then use the message transmission of joint tree, so as to improve the inference accuracy of uncertain events using Bayesian network. By inputting the employment data information of college students, individual information of college students, such as family environment and mastery of work skills, and the type data of college students' innovative employment security mechanism into the network model, we can obtain the relevance of college students' individual factors to the choice of innovative employment security mechanism and employment. The results show that individuals with higher education are more inclined to choose the policy of providing employment information, and they are easier to find a job. The lower the educational background and female college students are more inclined to the system and policy of job provision.

### 4.2. BP Neural Network Combined with Discrete Dynamic Modeling of Internet of Things to Construct the Evaluation Model of College Students' Innovative Employment Security Mechanism

#### 4.2.1. Experimental Data

In this experiment, we select the number of graduates from 50 colleges and universities in 2019 and the four most popular employment security policies for college students. The four policies are as follows: (i) provide employment information, (ii) provide labor security agency services, (iii) provide employment opportunities, and (iv) provide employment skills training. And the number of college students successfully employed after obtaining a certain policy as the sample data, as shown in Figure 4.

The figure above shows the statistics of college students' employment in recent years. It can be seen from the picture that with the increase in samples, a peak will appear every time a certain number is reached, as shown by the yellow dotted line in Figure 4.

#### 4.2.2. Result Analysis

100 employed samples are selected from the sample database, and the corresponding classification marks are made according to whether the samples accept four kinds of college students' innovative employment security mechanisms.

*(1) Determine the Analysis Sequence*. In this step, we need to calculate the factors reflecting all the characteristics of the whole system as the reference sequence and then get the factors affecting the system as the comparison sequence. Here, we take the employment number of college students as the reference series and the employment number of college students under different security systems as the comparison series.

*(2) Dimensionless*. Because the dimensions referenced by each factor in the system will be different, it will be difficult to compare, and the results will be error. Therefore, we need to deal with each factor dimensionless to make it a unified reference standard.

*(3) Obtain Correlation Coefficient*. Correlation degree is the degree of shape difference between data curves, which can also be regarded as the fitting degree between them. The difference between curves affects the magnitude of correlation degree and the difference in correlation coefficient *ρ* is the resolution coefficient. It has a negative correlation with resolution, *ρ.* The value range is between 0 and 1, usually 0.5.

*(4) Get Relevance*. The correlation coefficients of a system are different at different times, so there are multiple values of the coefficient. For the convenience of calculation and comparison, the average value of each point is used here.

*(5) Sort by Relevance*. Rank the correlation between four different employment security systems and college students' employment. The greater the correlation degree value indicates that the employment security system can better help college students obtain employment.

The calculation shows that among the four main college students' employment security mechanisms, the largest value is to provide employment information and then to provide jobs, employment skills training, and understanding labor security agency services. It can be concluded that among the employment security mechanisms, the one that has the greatest impact on the successful employment of college students is to provide employment information.

In addition, this article uses BP neural network algorithm to predict the number of college students after the implementation of college students' employment security mechanism, and the results are shown in Figure 5.

According to the figure, after importing the employment data of college students into BP neural network algorithm for training, the predicted employment number of graduates is roughly consistent with the actual data, but there is still a certain error, which is caused by the insufficient number of training samples.

## 5. Conclusion

This article mainly studies the historical development trend and discrete dynamic modeling and analysis technology of college students' innovative employment security mechanism under the background of the Internet of things. In this article, two different modeling methods, Bayesian network and BP neural network, are used to conduct discrete dynamic modeling on the influencing factors and employment security mechanism of college students' employment and find out four factors affecting college students' employment. Also get the main factors affecting college students' employment. In short, the formulation and improvement of employment security mechanism is a multidimensional and multilevel problem. Whether we can help graduates get employed smoothly is not only related to the type and implementation of the security mechanism but also closely related to the graduates' personal factors, family environment, and other factors. When formulating the employment security system for college students, the state should consider the factors such as regions, colleges, and universities and the working skills mastered by students and then analyze the specific problems. We will adjust employment security mechanisms and policies to achieve a balance between supply and demand in the talent market. This article has some innovative contributions, but there are still multidimensional and multilevel issues to discuss the formulation and improvement of employment security mechanism. Therefore, further research and analysis are needed in the future research.

## Figures and Tables

**Figure 1:** Bayesian network structure diagram.

**Figure 2:** Processing flow chart.

**Figure 3:** Result comparison chart.

**Figure 4:** Employment number of college students.

**Figure 5:** Projected employment figure.

## Data Availability

The data used to support the findings of this study are available from the corresponding author upon request.
